# Functional New Transcription Factors (TFs) Associated with Cervical Cancer

This article has been retracted.

**DOI:** 10.1155/2022/8381559

**Published:** 2022-01-25

**Authors:** Yicheng Jiang, Shi Chen

**Affiliations:** ^1^Department of Oncology, People's Hospital of Chongqing Hechuan, Chongqing, China; ^2^Department of Oncology, Chengdu Jinniu District People's Hospital, Chengdu, Sichuan, China

## Abstract

The goal of this research was to find noval transcription factors (TFs) that are involved in cervical carcinogenesis. The Gene Expression Omnibus (GEO) database was utilized to analyze ten cervical cancer datasets using the Robust Rank Aggregation (RRA) technique. Survival and differential expression were validated using GEPIA (Gene Expression Profiling Interactive Analysis). The transcriptional regulatory network and putative targets were built using Cytoscape. A real-time PCR (quantitative real-time polymerase chain reaction) experiment was used to confirm the mRNA expression. Using public cervical cancer single-cell RNA-sequencing (scRNA-seq), bulk TCGA-CESC RNA-seq, and microarray datasets, coexpression correlations between putative targets and TFs were confirmed. After combining the results of 10 datasets, 8 TFs, including EMX2 (Empty Spiracles Homeobox 2), were chosen among 385 robust DEGs. In the normal female reproductive tract, EMX2 is extensively expressed, but it is reduced in cervical cancer. Overexpression EMX2 suppresses the proliferation of HeLa cells. 12 potential targets of EMX2 were selected. Our research has revealed evidence that EMX2 acted as a tumor suppressor in cervical cancer and PDZRN3 might be possible target of EMX2 in cervical cancer. It might be a therapeutic target in the future.

## 1. Introduction

Despite the widespread screening programs, cervical cancer remains the third most common cancer in developing countries [1]. Based on the implementation of cervical screening programs with the referred adoption of improved screening methods in cervical cytology with the knowledge of the important role of the human papilloma virus (HPV), its incidence is decreased in the developed world [1]. Women in low- and middle-income nations were more prone to cervical cancer due to a lack of systematic screening and HPV (human papillomavirus) immunization programs [2, 3]. This malignancy has also put a great pressure on China's national health system. According to local CDC (Centers for Disease Control and Prevention) data, the incidence and fatality rate grew with time, notably in poor-living rural parts of the country's interior provinces, from 1991 to 2013 [4]. In 2018, this country accounted for more than 20% of all cervical cancer cases worldwide [5, 6].

Transcription factors (TFs) are becoming an increasingly attractive target for therapeutic intervention. In many malignancies, including cervical cancer, deregulated TFs play a role in the deregulation of oncogene and tumor suppressor genes. TFs are the major regulators of gene expression because they attach to the DNA promoter or enhancer regions of certain genes. TFs that have been mutated or unregulated facilitate abnormal gene expression, including the blocking of differentiation and cell death gene expression programs, as well as cancer's hallmark features [7, 8]. Most notably, homeobox-containing TFs, the master regulators in early embryological development and morphogenesis, are dysregulated in cervical cancer. Abnormal proliferation and aggressive behavior triggered by homeobox TFs could be observed in cervical cancer. MNX1 (Motor Neuron and Pancreas Homeobox 1) overexpression, for example, has been linked to cervical cancer advanced stages and lymph node metastases [9]. Overexpression of HOXC6 promotes cervical cancer cell cycle progression and proliferation via enhancing BCL2-mediated antiapoptotic effects [10], while PDX (pancreatic duodenal homeobox) has been shown to inhibit cervical cancer HeLa cell proliferation, invasion, and migration, enhance the overall health of tumor-bearing nude mice, and reduce tumor weight and volume [11]. In cervical cancer, LHX2 (LIM homeobox 2) is implicated in cisplatin resistance [12]. Under hypoxia, ZEB1 (zinc finger E-box binding homeobox 1) increases cervical cancer growth by recruiting tumour-associated macrophages that are reliant on CCL8 [13].

We used a bioinformatic methodology to identify DE-TFs (differentially expressed transcription factors) from cervical microarray datasets using the RRA (Robust Rank Aggregation) method in this work [14]. Differential expressions were further validated in GEPIA (Gene Expression Profiling Interactive Analysis) [15]. Among those DEGs, five homeobox-containing TFs (EMX2, HOXC6, ISL1, HOPX, and MSX1) were dysregulated in cervical cancer, indicating their particular involvement in cervical cancer tumorigenesis. Particularly, we focused on EMX2 (Empty Spiracles Homeobox 2), a tumor suppressor with limited reports in cervical cancer which is downregulated in cervical cancer. We showed that high expression of EMX2 is in normal female reproductive tract tissues but lost in cervical cancer. Overexpression of EMX2 in HeLa cells inhibits cell viability. More importantly, we constructed a transcriptional regulatory network of EMX2 and identified 12 potential targets of EMX2. Finally, we showed that EMX2 might be a direct upstream regulator of PDZRN3 (PDZ Domain Containing Ring Finger 3). Previous study showed it was a target of human papillomavirus type 16 (HPV-16) and HPV-18 E6 in cervical cancer [16]. Based on these findings, EMX2 may act as a tumor suppressor in cervical cancer and may be exploited as a potential therapeutic target candidate in the future.

## 2. Material and Methods

### 2.1. Microarray Dataset

We used microarray datasets with both normal samples and cervical primary cancer tissue (*n* > 5) after searching for “cervical cancer” as a keyword in the GEO (Gene Expression Omnibus) database.10 publicly available datasets including GSE166466 (not published), GSE29570 [17], GSE52903 [18], GSE55940 [19], GSE63514 [20], GSE63678 [21], GSE6791 [22], GSE7410 [23], GSE7803 [24], and GSE9750 [25] were downloaded from [26]. GSE67522 [27] and GSE151666 [28] datasets containing HPV infected cervical samples were also downloaded for further analysis.  Table 1 shows the detailed information for these GEO datasets.

### 2.2. Cell Line and Culture

Cervical cancer cell line HeLa were purchased from American Type Culture Collection (ATCC) and maintained in Central Laboratory of local hospital experiment center and maintained in high-glucose DMEM (Dulbecco's Modified Eagle Medium) with 10% FBS (Fetal Bovine Serum) plus 100 units of penicillin and 100 *µ*g of streptomycin and maintained in a humid incubator at 37°C in 5% CO_2_.

### 2.3. TCGA-CESC RNA-Sequencing Dataset

The TCGA-CESC (The Cancer Genome Atlas-Cervical Squamous Cell Carcinoma and Endocervical Adenocarcinoma) project's massive RNA-sequencing gene expression matrix was retrieved from the UCSC Xena project (http://xena.ucsc.edu) [29, 30]. The platform used in this assay was Illumina Hiseq Rnaseqv2 Platform and detected 308 samples with 20531 identifiers (version 2018-09-03). Also, the clinical information of these samples is obtained from corresponding TCGA-CESC curated survival (version 2018-09-03) and phenotype data (version 2019-12-06) and utilized in the study [31].

### 2.4. Robust Differentially Expressed Gene Analysis

The expression matrix from each microarray dataset downloaded from GEO was first automatically loaded into *R* statistical software (version 4.0.0, https://www.r-project.org/) using GEOquery package (version 2.58.0) and carried out quantile normalization and significance analysis with limma package (version 3.46.0). Subsequently, the candidates with adjusted *P* value less than 0.05 and |logFC| higher than 1 were regarded as significant DEGs in our RRA (Robust Rank Aggregation) method after integrating the results of 10 microarray datasets [14].

### 2.5. GEPIA Database Analysis

The GEPIA (Gene Expression Profiling Interactive Analysis) is an interactive web server containing the sequenced RNA expression data of 9736 tumors and 8587 normal samples from both the TCGA and GTEx (the Genotype-Tissue Expression projects) (http://gepia.cancer-pku.cn) [15]. Survival analysis in GEPIA2 for specific gene in TCGA-CESC dataset was also used.

### 2.6. Querying Transcription Factors from ENSEMBL Genome Databases

Annotated human TF gene list was obtained from the ENSEMBL human genome (GRCh38.p13) of European Bioinformatics Institute (EMBL-EBI) (http://www.ensembl.org/). The HGNC (HGO Gene Nomenclature Committee) symbols were filtered by the Gene Ontology (GO) Annotation using the term GO:0003700 for DNA binding transcription factor activities in order to get all the TFs. 1535 possible human TF genes were retrieved.

### 2.7. Transcriptional Regulatory Network Construction

Briefly, the predicted target genes from TFs were retrieved from the iRegulon [32]. The coexpressions between predicted target genes and TFs were validated in Pearson's correlation analysis in TCGA-CESC dataset by psych package in *R* with (|*r|* > 0.4 and *P* value < 0.05). The final transcriptional regulatory network was visualized in Cytoscape software (version 3.8.2).

### 2.8. Cell Transfection and Western Blot Analysis

Antibodies against *β*-actin (#TA811000S) and DDK (#TA50011-100) were purchased from OriGene (Beijing, China). Lipofectamine2000 (#11668027) was a product of Thermofish. Human EMX2 cDNA was cloned and inserted into pcDNA 3.1 mammalian expression-vector with a Myc-DDK tag (flag) in the C-terminal region for transient expression. HeLa cell transfection and western blot analysis were both performed according to the standard manual instruction.

### 2.9. Quantitative Real-Time PCR

Total RNA was extracted from the HeLa cell samples and the mRNA expression levels of EMX2, PDZRN3, COL14A1, MSX1, CXCL12, IGF1, ALDH1A2, SLIT2, PTGDS, AQP1, TGM1, SHCBP1, and MELK. The PrimerBank, a public resource for PCR primers, was used to design primers against the specific human target genes.  Table 2 shows the detailed primer information.

### 2.10. Cervical Cancer Single-Cell Transcriptome Analysis

10x genomic single-cell RNA-sequencing files of cervical cancer and normal tissue: GSE168652 (GSM5155196 and GSM5155197) were downloaded from NCBI GEO [33]. The expression matrix was loaded into *R* and analyzed by Seurat package (version 4.0.3) [34].

### 2.11. Dual-Luciferase Reporter Assay

Human PDZRN3 promoter upstream 2 kilobase sequence was obtained from human genomic DNA and inserted into pGL4 vector (PROMEGA). After transfection, dual-luciferase reporter assay was performed according to the standard manual instruction.

## 3. Results

### 3.1. Dysregulated Transcription Factors in Cervical Cancer

The expression profiles of cervical cancer tissues were compared with those of normal samples from 10 GEO cervical cancer datasets (GSE166466, GSE29570, GSE52903, GSE55940, GSE63514, GSE63678, GSE6791, GSE7410, GSE7803, and GSE9750) by the limma (linear models for microarray analysis) package in *R* statistical software. Following integration of 10 dataset results using the RRA (Robust Rank Aggregation) analysis, 385 robust DEGs (235 significantly upregulated and 150 significantly downregulated genes) were obtained, with adjusted *P* values of 0.05 and |logFC | >1 as the cutoff criterion. Then, DE-TFs were selected from the DEGs, to investigate the transcriptional misregulation in cervical cancer. A total of 8 TFs were among from 235 up DEGs, including E2F8 (*P* = 8.72*E* − 07, logFC = 1.227), FOXD1 (*P* = 8.36*E* − 15, logFC = 1.200), FOXM1*PP* = 1.25*E* − 17, logFC = 1.723), HOXC6 (*P* = 2.08*E* − 11, logFC = 1.372), IFI16 (*P* = 3.47*E* − 16, logFC = 1.136), MYBL2 (*P* = 9.28*E* − 13, logFC = 1.331), PLSCR1 (*P* = 8.31*E* − 17, logFC = 1.311), and STAT1 (*P* = 5.19*E* − 18, logFC = 1.314). Meanwhile, 12 other TFs from 150 down-DEGs were obtained, as AR (*P* = 6.57*E* − 20, logFC = −1.557), EMX2 (*P* = 1.82*E* − 09, logFC = −1.101), FOS (*P* = 2.00*E* − 12, logFC = −1.154), FOSB (*P* = 4.47*E* − 17, logFC = 1.559), HOPX (*P* = 1.13*E* − 13, logFC = −1.669), ISL1 (*P* = 7.73*E* − 13, logFC = -1.105), KLF4 (*P* = 3.27*E* − 16, logFC = −1.281), MSX1 (*P* = 4.84*E* − 14, logFC = −1.039), NDN (*P* = 6.43*E* − 15, logFC = −1.324), PEG3 (*P* = 4.82*E* − 11, logFC = 1.001), and PGR (*P* = 2.80*E* − 10, logFC = −1.260) along with ZBED2 (*P* = 9.06*E* − 09, logFC = −1.151). TFs like FOXM1, MYBL2, and STAT1 have been extensively studied in cancers including cervical cancer. The presence of sex steroid hormones receptor genes like AR and PGR might imply a unique transcriptional regulation for gynecological cancers.  Figure 1 shows that EMX2 is downregulated in cervical cancer.

Similar dysregulated expression patterns of most TFs were in cancer tissues from 306 samples of TCGA-CESC (The Cancer Genome Atlas-Cervical Squamous Cell Carcinoma) and 13 matched normal tissues from GTEx (Genotype-Tissue Expression) dataset validated in GEPIA (Gene Expression Profiling Interactive Analysis). Expressions of E2F8, FOXM1, FOXD1, HOXC6, MYBL2, PLSCR1, and STAT1 were significantly promoted in TCGA-CESC tumor tissues. On the other hand, AR, EMX2, KLF4, ISL1, NDN, MSX1, PEG3, and PGR were suppressed in cervical cancer (*P* < 0.05). However, no significance difference was identified between cancerous and matched normal tissues for IFI16, HOPX, ZBED2, FOS, and FOSB (*P* > 0.05).

### 3.2. Downregulation of EMX2 in Cervical Cancer and Suppression of Proliferation

Homeobox-containing genes were master players in morphogenesis and cell differentiation in animals, and their dysregulation would trigger great changes in cell fate determination. There were at least five homeobox-containing genes, EMX2, HOPX, HOXC6, ISL1, and MSX1, dysregulated in cervical cancer. In particular, we focused on EMX2 (Empty Spiracles Homeobox 2), an important morphogenesis regulator that has received little concern in cervical cancer research. The suppressed expression of EMX2 in cancer tissues from 306 samples of TCGA-CESC and 13 matched normal tissues from GTEx dataset was validated in GEPIA (Gene Expression Profiling Interactive Analysis) (*P* < 0.05). Meanwhile, EMX2 expression was significantly correlated with overall survival in the Survival Analysis Function provided by GEPIA 2 as a significant protective factor (hazard ratio < 1, *P* < 0.05). Pathological Stage Plot also indicated a loss of EMX2 in high AJCC (American Joint Committee on Cancer) pathological stage (*F* value = 1.76, Pr (>*F*) = 0.156). We constructed a mammalian expression-vector pcDNA 3.1 containing human EMX2 full-length CDS sequence. pcDNA 3.1 of Myc-DKK (Flag) EMX2 or an empty vector were both transfected into HeLa cells for 24, 48, and 72 hours. The MTT assay results indicated that HeLa cell viability was significantly affected in OE-EMX2 group after 24-, 48- and 72-hours' transfection (*P* < 0.05). These results indicated that EMX2 was downregulated in cervical cancer and may act as a tumor suppressor.

### 3.3. High Expression of EMX2 in Normal Female Reproductive Tract but not in Cancerous Tissues

We investigated the expression patterns of EMX2 in normal tissues from GTEx and Human Protein Atlas (HPA) consortium and found its dominant expression in normal female productive tract. The highest levels of EMX2 expression in GTEx were found in the uterus, endocervix, fallopian tube, and ectocervix (average read counts over 50). While its expression was lower in other normal tissues such as the liver, pancreas, and lung. Similarly, EMX2 was found mainly expressed in the endometrium and fallopian tube according to the data from HPA (average read counts over 50). Furthermore, an antibody detected EMX2 protein expression at a low level in the nucleus of glandular cells in cervical tissues from a 34-year-old female provided by HPA (HPA065294). Glandular cells are a type of mucus-producing cell found in the tissue that lines the inner part of the cervix. However, the EMX2 protein failed to be detected in samples of cervical cancer. This finding suggested that EMX2 may play a role in the morphogenesis of the normal emale reproductive tract. However, we demonstrated above that EMX2 mRNA expression was frequently lost in cervical cancerous tissues.

### 3.4. HPV Infection Associated with Reduction of EMX2 in Cervical Cancer

HPV (human papillomavirus) infection is an important risk factor for cervical cancer tumorigenesis. We also showed that HPV infection status also affects EMX2 mRNA expression status according to the dataset from GSE67522 and GSE151666. For GSE67522, a significant reduction of mRNA EMX2 expression occurred in both HPV-16 infected normal and cancerous samples compared to HPV negative histologically normal controls (logFC < −1, *P* < 0.05). Meanwhile, in GSE151666, uninfected cancer tissue exhibited a higher EMX2 expression comparing to those HPV infected samples (logFC < −1, *P* < 0.05). However, no difference between cancerous tissue infected by HPV-16/18 subtype and other HPV subtypes. These results implied that EMX2 gene expression might be directly affected after HPV-16/18 infection, but further experimental validation is still needed to explore the mechanisms.

### 3.5. Transcriptional Regulatory Network of EMX2 in Cervical Cancer

To construct a transcriptional regulatory network, we have downloaded a total of 1566 predictive target genes of EMX2 from the iRegulon plug-in at Cytoscape to build the transcriptional regulatory network of EMX2. The coexpression relationship of predicted target genes with mRNA expression level of EMX2 was subsequently validated in TCGA-CESC dataset by Pearson correlation using psych package (version 2.1.6) in *R*. When coefficient |*r*|>0.40 and *P*-value < 0.05, the candidate target genes were selected. The 147 coexpressed predicted target genes were either positively (*n* = 135) or negatively (*n* = 12) associated with EMX2 expression in TCGA-CESC dataset. Among the 147 coexpressed predicted target genes, 12 were found to be robust DEGs, which were then used to build the transcriptional regulatory network. There were 9 positively associated genes (COL14A1, MSX1, CXCL12, PDZRN3, IGF1, ALDH1A2, SLIT2, PTGDS, and AQP1) as red and 3 negatively associated genes (MELK, TGM1, and SHCBP1) as blue. In order to further validate these possible targets, we transfected HeLa cell with pcDNA3.1, either containing the full encoding sequence of human EMX2 (NM 004098.4) or an empty vector for 24 hours. Exogenous EMX2 protein expression has been confirmed using Myc-DDK (Flag) antibody. We then extracted the cDNA from each sample for subsequent quantitative reverse transcription PCR (RT-qPCR) assay. The relative expression of PDZRN3, MSX1, PTGDS, and MELK was significantly alternated after pcDNA 3.1 EMX2 was transfected. The results showed an increase in PDZRN3, MSX1, and PTGDS mRNA expression, while the expression of the MELK was reduced.  Figure 2 is the transcriptional regulatory network for EMX2 and target genes.

### 3.6. Identified PDZRN3 as a Potential Target of EMX2

Additionally, we used single-cell transcriptome dataset of GSE168652 (normal and cervical cancer sample) to validate the coexpression relationship between EMX2 and its potential targets. Following filtering, a total of 19477 cell expressing 20935 genes were obtained and used for subsequent single-cell transcriptome analysis. A total of 15 Seurat clusters were visualized in tSNE (t-distributed stochastic neighbor embedding) projection after dimensionality reduction using Seurat package (version 4.03) in *R*. The origins of the cells (normal as red or cancer as blue) were loaded into to tSNE plot and the results have shown that each sample has different distributions of cell clusters. We showed that EMX2 was dominantly expressed in cell clusters from normal samples, as we expected. Interestingly, PDZRN3 also have a very similar expression pattern like EMX2. Meanwhile, in the tSNE feature plot, MSX1 and PTGDS have the most similar expression patterns, but not for COL14A1, ALDH1A2, and AQP1. Negatively correlated genes such as MELK, TGM1, and SHCBP1 have very distinct expression patterns and are found primarily in cancer cell clusters. This is consistent with our rt-q-PCR results after EMX2 overexpression in HeLa cells. The violin plot for expressions of EMX2, PDZRN3, and marker genes like COL1A2, APOD, and ACTG2 shows that they are almost only expressed in normal smooth muscle cells and fibroblast cells. The positive coexpression correlations between EMX2 and PDZRN3 (*r* > 0.60, *P* < 0.05) was confirmed in bulk-RNAseq datasets like TCGA-CESC and GTEx as well as microarray datasets like GSE29570, GSE67552, GSE63678, and GSE9750. Also, the positive coexpression correlation was confirmed in HeLa cells after overexpression of EMX2. Finally, we used JASPAR, a database of transcription factor binding profiles, to predict potential high-score EMX2 binding sites in the 2.5 kilobase (kb) upstream from the human PDZRN3 promoter region (3p13). Site 1 was very close to the PDZRN3 TSS (transcriptional start site), while site 2 was l.5 kb upstream. According to the luciferase reporter assay, overexpression of EMX2 in HeLa cells resulted in a relative 4-6-fold increase in PDZRN3-promoter luciferase activity. However, EMX2 did not activate empty luciferase reporter vector in HeLa cells (data not shown). These findings suggested that EMX2 could act as a direct upstream transcription regulator of PDZRN3 in cervical tissues.  Figure 3 is the coexpression of PDZRN3 and EMX2 in cervical cancer single-cell transcriptome dataset GSE168652.  Figure 4 is the potential binding sites of EMX2 in PDZRN3 promoter region.

## 4. Discussions

Cervical cancer is the world's fourth most prevalent gynecological cancer [1]. Cervical cancer's molecular etiology is complicated, and the processes are yet unknown. We showed in this research that homeobox-containing genes such as MSX1, HOXC6, HOPX, ISL1, and EMX2 are among the dysregulated genes. Homeobox genes were an evolutionarily conserved family of transcription factors that played a key role in cell differentiation and morphogenesis. As a result, it is possible that dysregulated homeobox genes are linked to aberrant proliferation or other tumor features in cervical cancer. MSX1 has been discovered to regulate cell cycle and apoptosis via inhibiting Notch signaling [35].

We concentrated on EMX2 in particular. EMX2, like other homeobox-containing transcription factors, had a unique role in regulating anatomical development patterns. It was required for the morphogenesis of a variety of tissues, including the central nervous system [36–39], the pelvic girdle [40], and the female reproductive system, including the uterus [41]. EMX2 expression was also detected in the primordia of the reproductive and excretory systems during development [42]. EMX2 was also essential for female reproductive tract uterine development and endometrial programming (FRT). These findings corroborate what we discovered regarding EMX2 expression in GTEx and HPA. Endometriosis patients had abnormal endometrial EMX2 expression, which was mediated by altered HOXA10 expression [43]. Furthermore, a nonsense mutation in EMX2 has been suggested as a possible cause of uterine didelphys [44]. EMX2 has also been implicated in mammalian reproductive regulation by modulating endometrial cell proliferation [45].

Numerous papers have reported the tumor suppressive effect of EMX2 and its downregulation in various cancer types, which is consistent with our findings in cervical cancer. For example, EMX2 inhibited lung cancer cell growth and epigenetically silenced [46]. It has the potential to be employed as a prognosis marker for stage I lung SCC patients as well as a prediction marker for stage II/IIIA lung SCC patients undergoing adjuvant treatment [47]. Ectopic expression of EMX2 in gastric cancer was decreased by adenoviral administration [48]. Downregulation of EMX2 is a predictive factor for colorectal cancer disease-free and overall survival [49]. Because induced EMX2 expression prevented tumor growth in glioblastoma cells, suppression of EMX2 preserved tumorigenic potential in glioblastoma cells [50]. In endometrial cancer, EMX2 was found to be downregulated and linked with tumor stage, grade, and depth of myometrial invasion [51].

EMX2 has been shown to inhibit a number of cancer-related pathways, including PI3K/AKT [52] and Wnt/-catenin [53]. The Wnt/-catenin pathway is important for normal tissue morphogenesis as well as tumor development, including cervical cancer [54, 55]. The reinstatement of EMX2 in H1299 cells resulted in a reduction in WNT signaling-dependent transcription activity [46]. EMX2 suppresses proliferation and carcinogenesis in colorectal cancer cells by inactivating the Wnt/-catenin pathway [53]. Emx2 was also found to be a direct regulator of Wnt1 expression in the developing mammalian telencephalon in a mouse model [56]. Many verified Wnt/-catenin pathway regulators, including as SLIT2, PDZRN3, and SHCBP1, were also discovered in the transcriptional regulatory network [57–59]. We established PDZRN3 as a possible EMX2 target in cervical cancer. The morphogenesis regulator PDZRN3 and its family members are involved in cell differentiation [58, 60, 61]. Furthermore, in cervical cancer, HPV-18 E6-induced PDZRN3 degradation can lead to an increase in STAT5 activation [16]. Through PDZRN3, it would be interesting to see if EMX2 affects the Wnt/-catenin pathway and STAT5 in cervical cancer.

## 5. Conclusions

We established a regulatory network of TFs and their anticipated target genes in cervical cancer using bioinformatics analysis, demonstrating a different regulatory pattern of TFs. We also observed that EMX2, a homeobox-containing gene, may have a unique tumor suppressive role in cervical cancer. More experimental data will be needed to determine the specific involvement of EMX2 in the morphogenesis of cervical tissues and the tumorigenesis of cervical cancer.

## Figures and Tables

**Figure 1:** EMX2 is downregulated in cervical cancer. (a) Heatmap of 20 transcription factor genes (8 upregulated and 12 downregulated) generated using package pheatmap (version 1.0.12) in R (version 4.0.0) software according to *P* value. The number in each cell represents logarithmic fold change in each dataset calculated by the limma R package. Each row in the heatmap represents one gene and each column indicates one dataset. Red indicates upregulation and blue represents downregulation. (b) Gene Expression Profiling Interactive Analysis (GEPIA) was performed to validate the differential expression of transcription factor in cervical cancer samples compared with normal samples in TCGA and GTEx dataset. The expression level from GEPIA was presented as log_2_(TPM + 1). The boxplots were generated directly from GEPIA2 (Expression DIY, Expression on Box Plots). Red box was the cancer tissue group, gray was the normal tissue group, and asterisk represented *P* < 0.01. The dots represented expression in each sample. (c) GEPIA2 Survival Plots for EMX2 mRNA expression association with overall survival in TCGA-CESC. (d) Pathological Stage Plot for EMX2 expressions in different stage of TCGA-CESC samples. GTEx, Genotype-Tissue Expression; RRA, Robust Rank Aggregation; TCGA, The Cancer Genome Atlas; TPM, transcripts per million.

**Figure 2:** Transcriptional regulatory network for EMX2 and target genes. (a) The network of EMX2 and its 12 predicted robust DEGs identified by iRegulon (version 1.3) were downloaded and visualized in Cytoscape software (version 3.8.2). (b) Western blot results for EMX2 (myc-DDK tag) expression validated in HeLa cells after transfection for 48 hours. (c) The real-time qPCR validation of 12 predicted target genes of EMX2 in HeLa cells after transfection. The relative fold change expression of each gene was shown in the bar plot. CESC, cervical squamous cell carcinoma and endocervical adenocarcinoma; DE, differentially expressed; EMX2, Empty Spiracles Homeobox 2; qPCR, quantitative polymerase chain reaction; OE, overexpression; TCGA, The Cancer Genome Atlas.

**Figure 3:** Coexpression of PDZRN3 and EMX2 in cervical cancer single-cell transcriptome dataset GSE168652. (a) tSNE plot showing 15 major clusters. (b) tSNE plot with annotations according to sample origin. Normal as red and cervical cancer as blue. (c, d) Feature tSNE plots depicting EMX2 and PDZRN3 (SRY-Box Transcription Factor 2). The color bar from gray to purple indicated the changes of expression values from low to high. (e) Violin plot showed distribution similarities of EMX2 and PDZRN3 in single-cell clusters along with markers like ACTG2, COL1A2, and APOD. EMX2, Empty Spiracles Homeobox 2; PDZRN3, PDZ Domain Containing Ring Finger 3; tSNE, t-distributed stochastic neighbor embedding.

**Figure 4:** Potential binding sites of EMX2 in PDZRN3 promoter region. (a) The JASPAR logo for EMX2 binding motif. (b) The schematic diagram indicated two possible binding sites in 2.5-kilobase region of human PDZRN3 promoter. The nucleotide sequences were shown. (c) The relative luciferase activity of when pGL4-PDZRN3 and pcDNA-3.1 EMX2 were both transfected into HeLa cells. EMX2, Empty Spiracles Homeobox 2; PDZRN3, PDZ Domain Containing Ring Finger 3.

**Table 1:** Detailed information on GEO datasets used in this article was listed.

Dataset	Platform	Sample size	Country
GSE166466	GPL23126	Normal cervical epithelium (*n* = 7)	China
		HPV 16^+^ high-grade squamous intraepithelial lesion (*n* = 6)	
		HPV 16 cervical squamous cell carcinoma tissues (*n* = 7)	
GSE29570	GPL6244	Normal (*n* = 17)	Mexico
		Cervical cancer (*n* = 45)	
GSE52903	GPL6244	Healthy exocervix (*n* = 17)	Mexico
		Cervical cancer biopsy (*n* = 45)	
GSE63514	GPL6244	Reference controls (*n* = 25)	United States
		Tumors (*n* = 31)	
GSE63678	GPL570	Normal (*n* = 24)	United States
		CIN lesions (*n* = 76)	
		Cancer specimens (*n* = 28)	
GSE6791	GPL571	Normal cervical tissue (*n* = 5)	United States
		Cervical cancer tissue (*n* = 5)	
GSE7410	GPL1708	Healthy cervical tissue (*n* = 5)	Netherlands
		Early-stage cervical tumor (*n* = 40)	
GSE7803	GPL96	Normal squamous cervical epithelia (*n* = 10)	United States
		Invasive squamous cell carcinomas (*n* = 21)	
GSE9750	GPL96	Normal cervical epithelium (*n* = 24)	United States
		Primary tumors (*n* = 33)	

**Table 2:** Primers used for qPCR analysis.

Gene symbol	Forward	Reverse	Product size (bp)
EMX2	CGGCACTCAGCTACGCTAAC	CAAGTCCGGGTTGGAGTAGAC	107
PDZRN3	AGTGGTGCAGGTGTTGAGAAG	GTGATGTCGGTTTGGGTTCC	96
MSX1	ACACAAGACGAACCGTAAGCC	CACATGGGCCGTGTAGAGTC	382
CXCL12	ATTCTCAACACTCCAAACTGTGC	ACTTTAGCTTCGGGTCAATGC	88
IGF1	GCTCTTCAGTTCGTGTGTGGA	GCCTCCTTAGATCACAGCTCC	133
ALDH1A2	AGTGTTTTCCAACGTCACTGAT	AGTCTGAGTTATTGGCTCTTTCG	122
SLIT2	AGCTTAGACGAATTGACCTGAGC	CCGAAGGCAGTTTATCTTGTTGG	191
COL14A1	CTTGCACAGTATAGTGGTGACC	AGTCCTTGATCCTGCTTCTGG	177
PTGDS	CCAGGGCTGAGTTAAAGGAGA	CGTCATGCACTTATCGGTTTGG	101
AQP1	TAACCCTGCTCGGTCCTTTG	AGTCGTAGATGAGTACAGCCAG	113
TGM1	ATCATCGGCAAGTTTCAGTTCA	TCCCGTAGTAAATTCTCCCAGAC	190
SHCBP1	TGGCACACTAATGTGTTCAAGG	TCACAGAGGTATGGTTCAGCA	98
MELK	AACTCCAGCCTTATGCAGAAC	AACGATTTGGCGTAGTGAGTATT	167

## Data Availability

The simulation experiment data used to support the findings of this study are available from the corresponding author upon request.
